# The Effect of Physical Exercise on the Elderly's Anxiety: Based on Systematic Reviews and Meta-Analysis

**DOI:** 10.1155/2022/4848290

**Published:** 2022-05-09

**Authors:** Feilong Wu, Junling Zhang, Haiying Yang, Juan Jiang

**Affiliations:** ^1^Department of Physical Education, Xi'an Aeronautical University, Xi'an 710000, China; ^2^Traditional Chinese Medicine Department, Binzhou People's Hospital, Binzhou 256600, China; ^3^Nursing Department, Binzhou People's Hospital, Binzhou 256600, China; ^4^School of Martial Arts and Dance, Shenyang Sport University, 110102 Shenyang, China

## Abstract

**Purpose:**

Based on meta-analysis to explore the effect of physical exercise on relieving the anxiety of the elderly.

**Methods:**

The retrieval time was published in the domestic and foreign literatures on the effect of physical exercise on the anxiety of the elderly published from 2005 to 2021. The random effects model was used to evaluate the mean standard deviation of the scores of the intervention group on reducing the anxiety level of the elderly before and after the test. According to the inclusion and exclusion criteria, the articles were screened, quality evaluated, and data extracted, and the literature was meta-analyzed by RevMan5.3.

**Results:**

In meta-analysis and systematic review, 17 papers finally met the inclusion criteria. After sensitivity analysis, the random effects model (MD = 8.00, 95% CI (6.90, 9.10), *Z* = 14.23 (*P* < 0.00001)) and the fixed effects model (MD = 7.71, 95% CI (6.98, 8.43), *Z* = 20.72 (*P* < 0.00001)) show that physical exercise has a positive and significant effect on the anxiety of the elderly.

**Conclusion:**

Physical exercise plays an important role in reducing the anxiety of the elderly. Therefore, regular physical exercise can be regarded as part of the elderly pension plan, but more high-quality research is needed to further explore the impact of physical exercise on elderly anxiety.

## 1. Introduction

Aging is a necessary stage of human natural development, during which specific physiological, psychological, and social changes will occur [1]. That is, aging refers to spontaneous and gradual irreversible changes, and its physical and mental strength are obviously damaged or degraded [2]. The National Bureau of Statistics of China estimates that by 2050, more than one-third of China's population will be over 60 years old [3]. According to WHO estimates, by 2020, people over 65 will account for 20% of the world's population, and about 70% of them will live in developing countries. Many chronic diseases occur in the elderly, including cardiovascular diseases (such as hypertension and coronary artery disease), bone diseases (such as arthritis and osteoporosis), and mental disorders (such as anxiety and depression) [4, 5]. In particular, the loss of physical independence and chronic diseases, the reduction of activities and stimulation, loss of relatives and friends, changes in daily life environment, fear, etc. of the elderly make the elderly more prone to mental stress and psychological anxiety [6]. Anxiety is a mental state in which individuals experience nervousness, restlessness, and rubbing hands and feet in the absence of corresponding objective factors [7]. Studies have shown that 40 million adults in the United States suffer from anxiety, and as many as 57 million adults in China suffer from anxiety disorders. Anxiety has become a serious global public health problem [6, 8]. Therefore, early recognition and appropriate treatment can prevent these consequences from occurring. Aslankhani et al. believed that physical exercise is one of the most important, easiest, cheapest, and available treatment options for the elderly [9]. Reed and Buck believed that physical exercise not only enables different parts of the muscles to interact but also improves the daily life of the elderly and plays an important role in regulating physical and mental health [10]. According to Ruuskanen and Ruoppila, after analyzing the intensity and frequency of physical exercise in the elderly, the results showed that there was a significant relationship between the depression score of the elderly and the frequency and intensity of physical exercise [11]. Some scholars have found that physical exercise can alleviate the anxiety of the elderly, especially long-term adherence to low-intensity aerobic exercise can effectively reduce anxiety levels, thereby better improving the overall emotional state of exercisers [12, 13]. So far, there have been a large number of studies on physical exercise to relieve the anxiety of the elderly, but the results of the studies are not the same. Meta-analysis is used to respond to these research hypotheses and solve this problem. The research combs through small samples and the results before and after physical exercise intervention, conducts systematic evaluation and statistical analysis, comprehensively reflects the previous research results more objectively, and provides them to the society, clinicians, and people in need in a timely manner, and then, it is of great significance and value to promote and popularize real and effective physical exercise therapy for relieving anxiety levels. Therefore, this study is aimed at determining the effect of physical exercise on alleviating anxiety in the elderly through meta-analysis and systematic review.

## 2. Materials and Methods

### 2.1. Search Method

The study used “physical exercise, exercise, aerobic exercise, sports training, physical activity, etc. and elderly anxiety” as the Chinese key word to search in CNKI, Wanfang, and CQVIP, with “Physical exercise, Exercise, Aerobic exercise, Sports training, Physical activity, etc. and Elderly anxiety” are English keywords. Search in domestic and foreign databases of ISI, Scopus, PubMed, Cochrane Library, ScienceDirect, BioMed, Embase, and Web of Science, looking for documents from 2005 to July 2021, all relevant papers and references used in reports found in the search are manually reviewed to find other possible sources of information.

### 2.2. Inclusion Criteria

The study selected papers with the following characteristics for meta-analysis: (1) original research papers, (2) clinical trial studies, (3) full text availability, and (4) elderly people who investigated the correlation between physical exercise and anxiety.

### 2.3. Exclusion Criteria

Selected studies were evaluated more accurately. Repetitive studies, retrospective studies, incomplete data, studies using previous data, and studies where the sample did not select the elderly were all excluded from the meta-analysis. Finally, 52 studies were included in the fourth stage, the quality evaluation.

### 2.4. Data Extraction and Evaluation

The final paper that enters the meta-analysis process will have more than 2 reviewers extract data from the included literature list. The checklist includes the following fields: the title of the paper, the name of the first author, the year of publication, the location of the study, the average sample size before and after the intervention, the sample standard deviation before and after the intervention, and the type of intervention. The quality of the paper is evaluated according to the selected and related items in the CONSORT checklist; the selected items are research design, background and literature review, research location and time, results, inclusion criteria, sample size, and statistical analysis. Articles that meet 6 or 7 criteria are considered high-quality articles; articles with 2 or more and less than 2 criteria are considered medium- and low-quality articles, respectively [14]. In this study, 17 papers were classified as medium- or high-quality papers by meta-analysis and systematic review, and 35 low-quality papers were excluded.

### 2.5. Statistical Analysis

RevMan5.3 was used for meta-analysis. Given that the background of the research is the effect of physical exercise on the anxiety of the elderly, the mean and standard deviation are used to combine the results of various research work. Each study uses a standard difference index. The *I*^2^ index is used to investigate the homogeneity and heterogeneity between studies. The random effects model and the fixed effects model are used to combine the reported results and conduct a meta-analysis. According to the Cochrane system evaluation, when the *I*^2^ index is less than 25%, it is considered low heterogeneity, 25-75% is moderate heterogeneity, more than 75% is high heterogeneity, and *I*^2^ not greater than 50% indicates that heterogeneity can be accept. *P* ≤ 0.01 was considered statistically significant, and the degree of bias was assessed by a funnel chart.

## 3. Results

### 3.1. Search Flowchart

According to the Guidelines for the Preferred Report (PRISMA 2020) of the Systematic Review and Meta-Analysis, we systematically evaluated all relevant research literatures on the effects of physical exercise on the anxiety of the elderly. A total of 1,005 related documents were searched for the first time. After a systematic review of the documents, 17 research papers published from 2005 to July 2021 were finally included in the quantitative synthesis, which is the final evaluation (Figure 1).

### 3.2. Basic Characteristics and Quality Assessment

The 17 articles were finally included in the study for data statistics. There were 1151 subjects in the study, including 1022 in the experimental group and 1099 in the control group. Among the included evaluation documents, 12 were rated as high quality, and 5 were rated as medium.  Table 1 shows the basic characteristics and quality assessment of the final included studies. The characteristics of the risk of bias in the included studies were evaluated (Figure 2). As shown in the figure, most studies do not have a high risk of selection bias or do not report information about research selection, and only a few studies have a low or unclear risk of bias. Most studies (above 50%) have a low risk of bias, and more than half of the included studies use validated tools to measure the effect of physical exercise on elderly anxiety.

The results of the heterogeneity test reported by the meta-analysis show (see Figure 3) that there is high heterogeneity between studies (heterogeneity: *I*^2^ = 81%, Tau^2^ = 7.87, Chi^2^ = 85.55, df = 16, *Z* = 7.53, *P* < 0.00001). After applying sensitivity analysis, it is found that 8 articles are the root cause of high heterogeneity, including Asiachi-2017, Bethany-2-3-2005, Khesali-2018, Teixeira-1-3-2013, Xiao-2016, and Zhao-2015. After excluding the 8 groups of indicators, the fixed model and the random model were tested, and the results showed inconsistency (*I*^2^ = 38%, df = 8 (*P* = 0.11)), and the funnel chart showed that there was no publication bias (Figure 4). Meta-analysis results show that the random effects model (MD = 8.00, 95% CI (6.90, 9.10), *Z* = 14.23 (*P* < 0.00001)) (Figure 5) and the fixed effects model (MD = 7.71, 95% CI (6.98, 8.43), *Z* = 20.72 (*P* < 0.00001)) indicate that physical exercise has a significant effect on the anxiety of the elderly, which indicates that the test results are stable (Figure 6).

## 4. Discussion

The root cause of anxiety is people's inability to resolve conflicts in their minds, which leads to a large part of people's energy being spent on how to solve their psychological problems and further causes their psychological measurement incoordination, which will affect all aspects of life [26]. To this end, this study is aimed at determining through meta-analysis that physical exercise can effectively reduce or alleviate the anxiety state of the elderly. The results of the study showed that the anxiety level in the control group was very high, and there was a significant difference in the average scores of the elderly in the intervention group before and after the experiment on the severity of anxiety. Therefore, taking physical exercise intervention to change the original lifestyle of the elderly can better control the individual's anxiety level, prevent diseases, reduce other symptoms, and have a better impact on the physical and mental health of the elderly [26, 27]. Research results show that physical exercise can not only enhance cardiorespiratory health, increase muscle strength and endurance, and reduce physical fatigue but also promote communication and exchanges between people, release psychological pressure, and regulate emotional states and at the same time can overcome loneliness and cultivate. Psychological adaptability and other aspects play an important role [26, 28–30]. Physical exercise not only significantly improves the loneliness of the elderly but also plays a mediating role in the process of achieving happiness in the elderly [31]. A large number of research documents have found that physical exercise can reduce the level of anxiety and reduce the recurrence of anxiety after stagnant exercise, and it is also one of the important means to strengthen the physical and mental health of the elderly. Appropriate physical exercise can not only relieve negative mental states and induce positive mental states but also improve the loneliness, anxiety, depression, and happiness of the elderly [32–34]. A study by Camacho et al. found that people who regularly participate in sports will have a 1.5 times lower risk of depression and anxiety than people who do not participate in sports [8]. Some scholars found in their research that ballroom dancing had a significant effect on the anxiety regulation of the elderly before and after the intervention (*P* < 0.05). There was statistical significance between physical exercise and the psychological status of the elderly (*P* < 0.05) [35, 36]. Physical exercise is negatively correlated with psychological anxiety. Physical exercise can relieve the anxiety state of the elderly. The longer the physical exercise cycle, the lower the anxiety level of the elderly. At the same time, participating in physical exercise can effectively improve the respiratory system and cardiopulmonary function of the middle-aged and elderly people. It can effectively improve the lower limb balance ability and central system function of middle-aged and elderly people [37, 38]. Some scholars have found through experimental data that physical exercise can not only reduce and alleviate emotional disorders such as depression and anxiety but also positively delight the body and mind and maintain a positive and optimistic attitude, thereby reducing the incidence of depression and anxiety in the elderly [39]. Through a comparative analysis of the time, intensity, peers, and attitudes of physical exercise, it is found that the elderly who regularly participate in physical exercise have almost no depression and anxiety, and it is confirmed that physical exercise can effectively reduce the negative emotions of the elderly [40]. Research by Katula et al. believes that only one aerobic physical exercise can reduce the anxiety level of the elderly, thereby effectively improving the mental health status [41]. A study by Atashzade et al. found that 30 minutes of running can significantly improve the unhealthy state of mind, such as tension, fatigue, anxiety, depression, and anger, while maintaining a high level of energy [42]. Some studies have found that Health Qigong emphasizes the “three-regulation” holistic view of exercise, which can alleviate the stimulation of bad mental emotions on the brain, thereby improving the health of the human body and alleviating anxiety and depression levels [43]. Aerobic exercise has a significant effect on improving the physical fitness of participants and alleviating anxiety levels, and during the 12-week follow-up period after participating in exercise, the antianxiety effect of exercise continues to play a role [44]. The antianxiety effect of sports can be explained by a variety of mechanisms, including sports biology, medicine, physiology, and psychology. Biologically speaking, one of the main ways to improve physical health is to produce antianxiety effects through participation in sports, thereby affecting the level of neurotransmitters related to anxiety, reducing stress hormones, and reducing muscle tension after sports activities [45]. From the perspective of exercise physiology, physical exercise can increase stroke volume, drop in resting heart rate, and thicken myocardial fibers, thereby increasing myocardial contractility [46, 47]. From a psychological point of view, physical exercise can reduce anxiety by increasing the level of physical activity, strengthen the positive conditions of the reaction and adapt to changes in the external environment, and further improve the human body's ability to work and disease resistance [48].

## 5. Conclusions and Limitations

The research results show that physical exercise has a significant positive effect on the anxiety of the elderly. Physical activity and exercise are one of the most important, easiest, and cheapest treatments for anxiety disorders and have a positive effect on improving mental disorders in older adults. Regular exercise can effectively enhance cardiorespiratory fitness, increase muscle strength and endurance, reduce physical fatigue, improve morale, and improve the ability to perform daily tasks in older adults and was found to be greater in older adults. In addition, physical activity significantly affects and helps manage anxiety and improves overall health. Therefore, the regular exercise program can be regarded as a part of the pension plan and one of the means to improve the health service system for the elderly. It is to promote the combination of “physical, medical and nursing care” to promote healthy aging. One of the limitations of this study is that the survey results are affected by the mental state of the participants' answers or insufficient accuracy; the sample size is small, and the experimental observation time is short.

## Figures and Tables

**Figure 1:** Document selection flow chart.

**Figure 2:** Characteristics of risk of bias in included studies.

**Figure 3:** The effect of physical exercise on the anxiety of the elderly.

**Figure 4:** Funnel chart drawn by included studies.

**Figure 5:** The random effects model tests the effect of physical exercise on the anxiety of the elderly.

**Figure 6:** The fixed effects model tests the effect of physical exercise on the anxiety of the elderly.

**Table 1:** Basic characteristics and quality assessment of the included studies.

Author and publication time	Site	Practice sports	Sample size	Before intervention (mean ± SD)	After intervention (mean ± SD)	Quality assessment
Khesali, 2018, [15]	Iran	Tai chi	60	41.79 ± 9.5	29.41 ± 7.64	Higher
Asiachi, 2017, [16]	Iran	Yoga	30	73.6 ± 6.2	71.3 ± 7.5	Medium
Teixeira-1, 2013, [17]	Portugal	Physical activity scale	70	37.24 ± 13.48	34.6 ± 5.71	Higher
Teixeira-2, 2013, [17]	Portugal	Physical activity scale	70	46.68 ± 13.12	36.24 ± 8.82	Higher
Teixeira-3, 2013, [17]	Portugal	Physical activity scale	70	37.29 ± 9.12	37.45 ± 7.57	Higher
Teixeira-4, 2013, [17]	Portugal	Physical activity scale	70	46.48 ± 10.97	38.9 ± 8.15	Higher
Park, 2011, [18]	North Korea	Tai chi	23	50.55 ± 8.76	46.91 ± 14.33	Higher
Cassilhas, 2010, [19]	Brazil	Zhou resistance exercise	20	62.91 ± 1.3	56.13 ± 3.81	Higher
Bethany-1, 2005, [20]	USA	Yoga	11	35.64 ± 8.82	26.36 ± 8.59	Higher
Bethany-2, 2005, [20]	USA	Aerobic exercise	11	29.73 ± 8.78	29.0 ± 6.72	Higher
Bethany-3, 2005, [20]	USA	Walk	10	33.1 ± 8.94	32.5 ± 7.49	Higher
Antunes, 2005, [21]	Brazil	Endurance sports	23	40.78 ± 9.21	28.56 ± 5.5	Medium
Xiao, 2016, [22]	China	Health Qigong	108	35.78 ± 10.154	32.274 ± 8.194	Medium
Chen-1, 2016, [23]	China	Sports participation	64	51.31 ± 6.52	41.64 ± 5.672	Medium
Chen-2, 2016, [23]	China	Sports participation	265	51.48 ± 7.38	44.25 ± 5.33	Higher
Zhao, 2016, [24]	China	Health Qigong	186	36.86 ± 6.50	33.05 ± 6.49	Higher
Zhao, 2015, [25]	China	Fitness ballroom dancing	60	46.54 ± 5.24	39.29 ± 4.29	Medium

## Data Availability

The data used to support the findings of this study are within the article.
